# Advance in the Correlation between Diabetic Nephropathy and Abnormal Serum Thyroid Hormone Levels in Patients

**DOI:** 10.1155/2023/8947035

**Published:** 2023-05-08

**Authors:** Zhiqiu Liu

**Affiliations:** Jiangxi Medical College, Nanchang University, Nanchang, China

## Abstract

This study was developed to explore the correlation between diabetic nephropathy (DN) and abnormal serum thyroid hormone (TH) levels in patients, which can provide a reference for disease prevention and control in patients with DN. DN is the most serious complication of diabetes. The mortality rate of diabetic patients with DN is approximately 30 times higher than that of diabetic patients without DN. DN leads to high blood sugar, which causes vascular dysfunction in patients, causes cardiovascular disease, aggravates the disease and disease complexity, and thus increases the mortality of patients. DN patients often have oxidative stress and even fibrosis in severe cases. TH has a potential renal protective effect and can also regulate glucose metabolism and improve abnormal glucose tolerance and insulin resistance. Abnormal serum TH levels increase the risk of DN. Normal thyroid function plays an important role in regulating the physiological functions of the human body. Hormonal disorders promote the development of diabetes mellitus (DM) into DN. The pathogenesis, clinical manifestations, detection, and treatment methods of DN were reviewed in this study. The research progress of the influence of TH on DN was analyzed. This study is conducive to clinical research on DN and provides a reference.

## 1. Introduction

Diabetes is a chronic disease with a high incidence and can cause great suffering to patients. With changes in people's diet and exercise habits, many people are used to a high-fat and high-salt diet, and exercise time is less, resulting in an increasing number of diabetes mellitus (DM) patients. Diabetes generally occurs in middle-aged and elderly people. In recent years, the age range of DM onset has also expanded. Many young people also develop DM, endangering their lives and health [1]. Diabetes can seriously affect people's normal lives and change their eating habits. Diabetes is affected by age, sex, race, lifestyle, and living environment. The common clinical manifestations of diabetic nephropathy (DN) are proteinuria and hematuria, as well as hypertension and impaired renal function (RF), which complicate the patient's condition and make the disease more difficult to cure. Patients with advanced DN will also have renal failure, which seriously affects the normal physiological function of patients and will greatly improve the mortality of DM patients. Patients with DM are prone to a variety of complications in the later stages, among which the incidence of DN is high, which has a great impact on patients [2]. The condition of DN is complicated, the condition is prolonged, and treatment is difficult. Patients will be repeatedly admitted to the hospital, causing a serious burden to social medical resources and families. The treatment of DN will aggravate the disease and be irreversible. Therefore, early detection and treatment are of great significance.

At present, the diagnostic methods of DN mainly include renal puncture tests, serological tests, ultrasound tests, and urinary microalbumin. Renal puncture examination has the advantages of high accuracy and a more accurate diagnosis of the disease. It is the gold standard for the detection of DN and is widely used in clinical practice. However, this kind of operation causes damage to the patient's body and brings pain to the patient, and the patient's acceptance is low. Serological tests have the advantages of easy operation, no exposure to radioactive substances, and good diagnostic effects. It has unique value in the examination and diagnosis of DN and has become a commonly used research method. Ultrasound examination is a common organ examination method in the clinic and is a standard imaging technique in diagnosis. It can observe the structure and function of lesions in real time, and it is simple, noninvasive, and easy to repeat. Thus, it has become an important tool for the early identification of disease types and etiology and has positive value in organ diagnosis and disease assessment. DN is refractory and difficult to treat in the clinic. Its mortality and disability rates have remained high for many years.

Thyroid hormone (TH) affects the growth and development of the kidney and can have a certain effect on the blood sugar of patients. The mechanism of thyroid action is combining with receptors to form a hormone receptor complex, which induces gene transcription and has a negative feedback regulation mechanism. Overproduction of THs will in turn suppress the hypothalamus and pituitary glands, to reduce hormone production. TH can promote metabolism, accelerate substance conversion, generate heat, and maintain normal body temperature. TH can also promote physical and intellectual development, has a significant impact on the nervous system, bone, and reproductive system, and can improve the nervous system, especially sympathetic nervous system excitability, so that human activity is maintained in a certain range. The synthesis process of TH consists of three processes. The first step is the uptake and transport of iodine and the thyroid acinar cell membrane has an iodine pump that has a strong ability to absorb and concentrate iodine. The second step is iodine activation and chloramiodization. The ingested iodine is oxidized by peroxidase into activated iodine in the microvilli at the top of the acicular epithelial cells. The activated iodine is then combined with thyroglobulin, and the tyrosine residues in the molecule are combined to form monoiodotyrosine and diiodotyrosine. The third step is the coupling process. Under the action of peroxidase, one molecule of monoiodotyrosine and one molecule of diiodotyrosine are coupled to T3, and two molecules of diiodotyrosine are coupled to T4. Under the action of proteolytic enzymes, thyroglobulin is further coupled and degraded, releasing T3 and T4 into the blood. TH is associated with DN [3]. At present, the clinical relationship between TH levels and DN is not clear, and research on this aspect is relatively rare. The clinical value of this study is that it explored the correlation between DN and abnormal serum TH levels in patients and provided a clinical reference for the influence of TH on blood glucose and renal function in patients with diabetes.

## 2. Advances in DN

### 2.1. Pathogenesis of DN

Diabetes is a very common disease with a high incidence and complicated complications. DN is more likely to occur in DM patients and is affected by many factors. The main influencing factors include genetics, abnormal blood glucose levels, and disorders of blood glucose metabolism, abnormal hemodynamics, and inflammatory stimulation [4]. DN has obvious heritability. Patients with a family history of DN have a greatly increased chance of DN. Genetic susceptibility and polymorphism play an important role in DN. The angiotensin converting enzyme gene increases the risk of DN. Abnormal blood glucose levels, which lead to metabolic disorders of the body, will also greatly increase the probability of DN. Many studies have shown that the activity of the polyol pathway can affect the incidence of DN [5, 6]. Elevated blood glucose in patients will increase the rate-limiting enzyme activity of the polyol pathway and affect the kidney function of patients. Changes in the structure of the basement membrane of the glomerulus can lead to sclerosis of the glomerulus, which makes patients prone to DN. Protein kinase C is a protein kinase involved in intracellular signal transduction and can be involved in the regulation of cell proliferation, differentiation, and apoptosis. High blood glucose levels in patients may lead to protein kinase C transmission pathways that stimulate cells to produce large amounts of protein kinase C, leading to increased glomerular damage in patients. Oxidative stress is also associated with DN. The inflammatory response plays a crucial role in the development of DN. Inflammatory cells infiltrate into the kidney, leading to increased release of inflammatory factors, resulting in glomerulosclerosis, interstitial fibrosis of renal tubules, and serious impact on the normal function of the kidney [7, 8].  Figure 1 shows the influencing factors of DN.

### 2.2. Stages and Clinical Manifestations of DN

DN is often accompanied by microangiopathosis of other organs or systems. DN is graded into the following five stages: I, glomerular hyperfiltration and renal hypertrophy, and this initial stage without histopathological injury; II, normal albuminuria phase, with GFR higher than normal level, and renal pathology showed thickened GBM, increased mesangial matrix, and increased urinary albumin excretion rate (UAE) after exercise (>20 *μ*g/min) and returned to normal after rest; III, early DN, also known as “persistent microalbuminuria,” the GFR begins to decline to normal, renal pathology shows glomerular nodular lesions and arteriolar hyalinosis, microalbuminuria, and the patient's blood pressure increases significantly; IV, clinical DN, with typical K-W nodules pathologically, and patients with persistent massive albuminuria are prone to nephrotic syndrome, and GFR continues to decline [9]; and V, end-stage renal failure, in which urinary protein is reduced due to glomerulosclerosis and the symptoms of uremia are obvious.  Figure 2 shows the stages of DN.

### 2.3. Diagnostic Methods for DN

1. Urinary microalbumin detection is a common method for the diagnosis of DN. This method has little harm to patients, a simple operation, a low price, and high acceptance of patients [10]. However, this method has strong limitations, such as having accurate diagnostic value only for some patients with DN, and has a good effect on the early diagnosis of DN.  Figure 3 shows the characteristics of urinary microalbumin detection.
2. Renal biopsy is the gold standard for the diagnosis of DN [11]. This detection method has high accuracy and specificity and has positive clinical value. However, this method can cause damage and pain to patients.  Figure 4 shows a schematic diagram of a renal needle biopsy.
3. For serological tests, there are more serological indicators in the diagnosis of DN, and patients have more selectivity. Serum cystatin C and *β*2 microglobulin have better diagnostic effects. Cystatin C can significantly reflect the filtration function of glomeruli, and it is easy to operate and highly acceptable to patients.  Figure 5 shows the serological indicators of DN.
4. Ultrasonic detection is easy to perform, noninvasive, and simple, and the results can be displayed quickly, which has important value for the evaluation of DN. Ultrasonic detection methods mainly include color Doppler ultrasound, contrast-enhanced ultrasound, and ultrasonic elastic imaging [12].  Figure 6 shows the ultrasonic detection method of DN.

### 2.4. Treatment of DN

1. *Blood Sugar Control*. Blood sugar is the most important factor affecting the development of the disease in patients with diabetes. Controlling blood glucose is of great significance to prevent DN. The main way to control blood sugar is by taking hypoglycemic drugs. It is necessary to select the most suitable drug for patients to control blood glucose. Patients with mild to moderate DN can choose gliquidone as a hypoglycemic drug, and patients with severe DN can receive insulin therapy [13]. Studies have found that treatment with L-lysine can slow the progression of DN [14].  Figure 7 shows the method of blood glucose control in DN.
2. *Blood Pressure Control*. Blood sugar and blood pressure are related to a certain extent, and abnormal hemodynamics may lead to abnormal blood sugar levels [15]. Reasonable control of blood pressure can effectively control the occurrence of DN. Angiotensin-converting enzyme inhibitors can control hypertension and have a positive protective effect on the kidneys.  Figure 8 shows the method of blood pressure control in DN.
3. *Lipid Contro*l. Hyperlipidemia can aggravate diabetes not only causing damage to pancreatic beta cells but also promoting glomerular and tubule interstitial fibrosis. Statins have good lipid-regulating effects; among which atorvastatin has good renal protection function and can promote the reduction of blood lipid levels in patients.  Figure 9 shows the methods of lipid control in DN.
4. *Anti-Inflammatory Therapy*. Inflammation can greatly aggravate the development of DN, so anti-inflammatory therapy is necessary [16]. Aldose reductase inhibitors act on the polyol pathway, preventing the conversion of glucose to sorbitol. The aldose reductase inhibitor epalrestat can significantly reduce the inflammatory response in DN patients. In addition, rosiglitazone, a common insulin sensitizer, has a positive anti-inflammatory effect.  Figure 10 shows the anti-inflammatory treatment of DN.
5. *Western Medicine Therapy*. Western medicine therapy has positive application value in the treatment of DN. The most common treatments are hemodialysis and peritoneal dialysis. Hemodialysis has a good blood purification effect and can significantly and effectively improve patients' blood conditions [17, 18]. Peritoneal dialysis also has a good clinical effect in the treatment of DN, and it is widely used in the clinic. Sodium-glucose cotransporter 2 (SGLT2) inhibitors have been shown to reduce the risk of major cardiovascular events and the probability of kidney disease in patients with type 2 diabetes. Changes associated with SGLT2 inhibitors have important effects on cardiorenal protection [19].
6. *TCM Treatment*. TCM also plays an important role in the treatment of DN. In the treatment of DN, prescriptions such as nourishing qi and nourishing yin are frequently used. The selection of traditional Chinese medicine for nourishing qi and nourishing Yin has positive application value in the prevention and treatment of DN. Because of its multitarget function, Chinese medicine has good clinical efficacy as the main or alternative therapy for DN. TCM and its bioactive ingredients have good clinical efficacy in the treatment and management of DN. Traditional Chinese medicine prescriptions also have the characteristics of treating both symptoms and root causes, safety and reliability, and few side effects, which can greatly improve the physique and condition of patients.  Figure 11 shows the characteristics of TCM treatment of DN.

### 2.5. Overview of TH Levels

TH is a hormone containing tyrosine condensation synthesized by thyroid follicular epithelial cells that can promote growth and development, regulate metabolism, and affect the physiological functions of various organs [20, 21]. THs include total T3, total T4, free T3, and free T4. Total T3 and total T4 are formed after the combination of TH and protein. Free T3 and free T4 play the role of TH in the blood. When free T3 and free T4 are exhausted, total T3 and total T4 shed proteins and become free THs again [22]. Thyrotropin activates the second messenger pathway, affecting the expression and release of some genes. TH-releasing hormone is composed of glutamic acid, histidine, and proline, and its secretion is affected by TH. Thyrotropin-releasing hormone is released from the hypothalamus and sent free to the anterior pituitary gland, where it binds to the thyrotropin-releasing hormone receptor to promote the release of thyrotropin [23, 24]. TH is regulated by thyroid stimulating hormone (TSH). TSH is a glycoprotein secreted by the anterior pituitary alkalophilic cells, released by the pituitary gland and free to the thyroid gland and the thyroid stimulating hormone receptor, which binds in the thyroid cells to activate the second messenger pathway and promote the expression of T3 and T4 genes.

## 3. Research Progress on the Relationship between TH Levels and DN

### 3.1. Effects of TH Levels on the Kidney

The kidney is an important organ affecting human growth and development, and its metabolism is regulated by TH levels. THs can activate the renin-angiotensin-aldosterone system, which has an important influence on hemodynamics [25]. TH affects the size, volume, and structure of the kidney to a certain extent. TH also has a regulatory effect on the blood circulation of the kidney. Peters et al. [26] explored the prevalence of TH abnormalities in patients with kidney disease and studied the relationship between serum levels of free triiodothyronine (FT3), thyroid stimulating hormone (TSH), and free thyroxine (fT4) and RF and proteinuria. The results found that among a large number of hospitalized patients, low triiodothyronine syndrome was 2.5 times more common in patients with advanced kidney disease than in those with normal RF. In patients with advanced CKD, both eGFR and proteinuria are closely related to THs. Close screening for thyroid status in patients with CKD at any stage, especially in patients with proteinuria, has positive clinical significance. The relationship between proteinuria and thyroid function in patients with chronic kidney disease is still controversial. Reinhardt et al. [27] studied the relationship between kidney and thyroid function in patients with negative thyroid antibodies among all patients with chronic kidney disease. The rT3 concentration was negatively correlated with proteinuria, and the level of rT3 was much lower in patients with severe proteinuria than in patients with mild or moderate proteinuria. The severity of proteinuria had no effect on TSH, FT4, T3, FT3, or TBG. EGFR was associated with increased T4, FT4, T3, FT3, and TBG, but not rT3. This suggests that the severity of proteinuria is inversely associated with rT3 in patients with thyroid antibody-negative chronic kidney disease. Hypothyroidism and hypofree triiodothyronine (FT3) syndrome (normal low FT3 levels of thyroid stimulating hormone (TSH)) are associated with cross-sectional reductions in RF in patients with chronic kidney disease (CKD) who have a severely reduced estimated glomerular filtration rate (eGFR) or end-stage renal disease (ESKD). Schultheiss et al. [28] evaluated the relationship between thyroid and RF and eGFR (cross-sectional) as well as renal events and mortality in CKD patients with mildly to moderately reduced RF. Patients with mild-to-moderate CKD with thyroid dysfunction were found to be at increased risk of adverse renal events and all-cause mortality over time. In contrast to TH (TH) 3,3′,5-triiodothyronine (T3) and thyroxine (T4), the current literature on TH metabolite concentrations in hypothyroidism and hyperthyroidism states is unclear. Jongejan et al. [29] studied the changes in 9 TH and its metabolites (THM) in a group of patients treated with DTC under different thyroid states and studied three potentially important determinants of THM concentration. All THMs were found to be markedly lower in hypothyroidism and higher in subclinical hyperthyroidism than in normal thyroid conditions. T3 concentrations remained within the reference range, and RF was associated with lower 3-monoiodothyronine (3-T1) concentrations. Thyroid function may be a factor affecting RF in the general population. Renal and thyroid function change with age. Thyroid function and RF decrease in elderly individuals. Wei et al. [30] evaluated the relationship between normal-range thyroid function and age-related decline in RF in elderly individuals. There is a notable correlation between RF and thyroid function, especially FT3, in elderly individuals. Clinicians may need to pay more attention to RF assessment and follow-up in older adults with low normal FT3 and high normal TSH.  Figure 12 shows the effect of TH levels on the kidney. These studies suggest that TH levels play an important role in kidney function, and abnormal hormone function may impair normal kidney function. Abnormal thyroid function may induce abnormal renal function, but the root cause of impaired GFR remains unclear. THs have a significant effect on blood pressure (BP) and kidney function because they affect glomerular filtration rate (GFR), and measures need to be taken to maintain healthy blood pressure and prevent the early development of kidney disease. Alsulami et al. [31] discussed the relationship between blood pressure, glomerular filtration rate, and thyroid-stimulating hormone (TSH) level in hypothyroidism patients and found that there was no correlation between blood pressure and TSH, while creatinine was directly correlated with TSH, and GFR was negatively correlated with TSH. Physicians in patients with hypothyroidism should aim to follow up on renal function to prevent premature complications.  Figure 12 shows the effect of TH levels on the kidney.

### 3.2. Effects of TH Levels on Blood Sugar

THs can control glucose uptake, glycolysis, and lactate transport and effectively regulate cellular glucose metabolism. Decreased TH sensitivity is a common phenomenon in the general population and may be related to metabolic parameters [32]. Mehran et al. [33] evaluated the cross-sectional correlation between TH sensitivity and DM, metabolic syndrome (MetS), and its components. A new thyroid feedback quantile index (TFQI), an indicator of decreased TH sensitivity, was found to correlate population variation with DM and hypertension in people with normal thyroid function. Eckert et al. [34] evaluated the relationship between thyroid autoimmunity in adolescents and young adults with type 1 DM and found that thyroid function was substantially suppressed in patients with DM. There is a certain relationship between thyroid function and DM. Birck et al. [35] studied thyroid stimulating hormone (TSH), free thyroxine (FT4), free triiodothyronine (FT3), their conversion rate (FT3: FT4), and the risk of DM in subjects with normal thyroid and patients with subclinical thyroid dysfunction. TSH, FT4, FT3, and FT3: FT4 ratios were not found to be associated with the development of DM. Using continuous variables; a 1-unit (1-U) increase in FT4 reduced DM risk, whereas a 1-U increases in the FT3: FT4 ratio increased DM risk. Increased 1-U of FT3 is associated with an increased risk of DM. These findings suggest that FT4 and FT3 levels and conversion rates may be additional risk factors associated with DM. Gu et al. [36] discussed the relationship between thyroid function and blood glucose in DM patients. It was found that a decrease in free TH levels was associated with an increase in blood glucose. After clinical treatment, the improvement in blood glucose and insulin resistance was accompanied by the recovery of hyponormal thyroid function. Chen et al. [37] evaluated the difference between T2DM patients with normal thyroid function and patients with abnormal TH. In T2DM patients with normal thyroid function, the FT3 level was positively correlated with SMI and negatively correlated with EWF, while the FT4 level was positively correlated with BFM and LLLMM. Thyroid function can influence body composition in T2DM patients with normal thyroid function. Although the incidence of thyroid dysfunction and diabetes is high in the general population, further research is needed to determine whether their interaction may be driven by other mechanisms, such as genetic predisposition.

### 3.3. Effect of TH Level on DN

The early stage of DN may present as a secondary nephrotic syndrome. The main clinical features of nephrotic syndrome are urinary protein loss and decreased serum albumin. Urinary protein contains thyroid-binding globulin, thyroxine carrier protein, prealbumin, and albumin. Normal thyroid function can protect against RF and prevent the occurrence of DN. Changes in TH levels are related to the pathogenesis and treatment of DN. Yang et al. [38] explored the relationship between THs and the risk of DN progression and selected the urinary albumin/creatinine ratio (ACR) and glomerular filtration rate (eGFR) to evaluate persistent proteinuria and staged chronic kidney disease. Compared with the nondiabetic kidney disease (DKD) group, the DKD group had higher levels of thyroid stimulating hormone (TSH) and lower levels of free triiodothyronine (FT3) and free thyroxine (FT4). The prevalence of thyroid dysfunction in the DKD group was drastically higher than that in the non-DKD group. The level of FT3 decreased gradually with the deterioration of DKD, and the level of TSH increased with the increase in KDIGO. FT3 and FT4 levels were negatively correlated with serum creatinine levels and ACR and positively correlated with eGFR. In contrast, TSH was positively correlated with ACR and negatively correlated with eGFR. Low FT3 levels were found to be an independent risk factor for DKD and DKD progression. Serum uric acid is associated with the progression of DN. THs regulate metabolism and insulin resistance. The relationship between SUA and thyroid function in patients with DKD is uncertain. Feng et al. [39] studied the relationship between thyroid stimulating hormone (TSH) and SUA in type 2 DM patients with early DKD. Compared with the normal SUA group and the control group, the SUA level in the high SUA group was increased, and the TSH level was decreased. There was no great difference in SUA and TSH between the normal SUA group and the control group. In type 2 DM patients with early DKD, TSH is negatively correlated with SUA. Decreased TSH is an independent risk factor for hyperuricemia in type 2 DM patients with early DKD. These results suggest that THs, especially TSH, may be involved in regulating uric acid metabolism in patients with early DKD. Thyroid autoantibodies can better detect thyroid function and have a positive clinical value. Thyroid peroxidase antibody (TPOAb), thyroid globulin antibody (TgAb), and thyroid-stimulating hormone receptor antibody (TRAb) are common thyroid autoantibodies. In diabetic patients, thyroid autoantibodies have a high sensitivity. In DN patients, FT3 and FT4 concentrations are decreased, while TSH levels are increased.

## Figures and Tables

**Figure 1:** Factors influencing DN.

**Figure 2:** Stages of DN.

**Figure 3:** Characteristics of urine microalbumin detection.

**Figure 4:** Schematic diagram of renal needle biopsy.

**Figure 5:** Serological indicators of DN.

**Figure 6:** Ultrasonic detection of DN.

**Figure 7:** Methods of glycemic control in DN.

**Figure 8:** Methods for blood pressure control in DN.

**Figure 9:** Methods for lipid control in DN.

**Figure 10:** Anti-inflammatory treatment of DN.

**Figure 11:** Characteristics of traditional Chinese medicine treatment of DN.

**Figure 12:** Effects of TH levels on the kidney.

## Data Availability

The data used to support the findings of this study are included within the article.

## Additional Points

*Summary and Prospect. *The incidence of DN is high, the treatment is difficult, the complications are many, and it seriously threatens the normal life of patients. Abnormal blood sugar and damage to renal function will aggravate the disease and increase the mortality of patients. TH plays an important role in the renal function of the human body and plays a certain regulatory role in the blood sugar level of the human body. Abnormal TH can aggravate diabetes, which can cause and aggravate DN. Hence, it is of great significance to maintain the stability of TH and make thyroid function play a normal role in the control and treatment of DN. This study reviewed the internal relationship between DN and TH levels, which provides a theoretical basis for the prevention, control, and treatment of DN patients. Nevertheless, the deficiency of this study is that there is no clinical verification. The principle of blood gas variation differences under DN has not been fully elaborated. In the future, verification and analysis can be carried out in clinical cases to further explore blood gas variation differences under DN to provide a reference for the clinical treatment of DN.
